# Integrative Analysis Reveals a Nine TP53 Pathway-Related lncRNA Prognostic Signature in Endometrial Cancer

**DOI:** 10.1155/2022/5432806

**Published:** 2022-10-10

**Authors:** Ying Wang, Xiaoling Qu, Lisha Li, Deng He

**Affiliations:** ^1^Department of Nursing, Tongji Hospital, Tongji Medical College, Huazhong University of Science and Technology, No. 1095 Jiefang Avenue, 430030 Wuhan, China; ^2^Department and Institute of Urology, Tongji Hospital, Tongji Medical College, Huazhong University of Science and Technology, No. 1095 Jiefang Avenue, 430030 Wuhan, China; ^3^Department of Obstetrics and Gynecology, Tongji Hospital, Tongji Medical College, Huazhong University of Science and Technology, No. 1095 Jiefang Avenue, 430030 Wuhan, China

## Abstract

**Background:**

TP53 mutation is a common mutation gene in uterine corpus endometrial carcinoma (UCEC), and the TP53 signaling pathway plays an essential role in the tumorigenesis, progression, and immune infiltration in UCEC. We aimed to discover TP53 pathway-related lncRNAs in UCEC. *Materials and methods*. 528 UCEC patients with 587 transcriptional profiles were enrolled in this study. We first investigated the differential status of TP53 signaling pathway between tumor and normal tissues by GSEA analysis, then identified TP53 pathway-related lncRNAs, accordingly establishing a nine TP53 pathway related to the lncRNA signature in the training set and verified this signature in the test set. Besides, the interaction network was constructed; the immune infiltration, drug response to cisplatin and paclitaxel, and mutation atlas were investigated. Finally, we performed a subgroup analysis to check the universality of this signature.

**Results:**

A nine TP53 pathway-related lncRNA prognostic signature was constructed and verified superior accuracy in predicting the overall survival of UCEC patients. Besides, high-risk patients showed a poor prognosis, but they were more sensitive to the cisplatin and paclitaxel. Notably, M2 macrophages were higher infiltrated in high-risk patients, and TP53 showed a significantly higher mutation in high-risk patients than low-risk patients.

**Conclusions:**

We constructed and verified a nine TP53 pathway-related lncRNA prognostic signature in UCEC, which also contributes to the decision-making of the chemotherapy.

## 1. Introduction

TP53 is one of the most significant genes in nearly all tumor types that are mutated in more than 50% of human cancers [1, 2]. It encodes p53 tumor suppressor protein, which mainly contributes to protecting the DNA integrity of the cells [3, 4]. As a protein encoded by the tumor suppressor gene, p53 protein can limit the proliferation of abnormal cells. It can limit tumor development through cell stress sensors, which can respond to DNA damage, hypoxia, oncogene expression, nutritional deprivation and ribosome dysfunction, and limit cell proliferation under these adverse conditions [5, 6]. In addition, p53 can respond to DNA damage and promote apoptosis or cellular senescence [7]. Under the condition of low-level stress, p53 can trigger protective survival-promoting responses, such as temporary cell cycle arrest, DNA repair, or production of antioxidant proteins, to maintain the integrity of the genome and repair the vitality of damaged cells [4]. Therefore, the TP53 signaling pathway plays a very important role in the normal life activities of cells [2]. In recent years, researchers are also committed to finding new potential regulatory genes related to the TP53 signaling pathway, especially long-chain noncoding RNA [8–10].

Long noncoding RNA (lncRNA) refers to noncoding RNA with a length of more than 400 nucleotides, including long intergenic no-coding RNA (Linc RNA) and natural antisense transcripts (NAT) [11, 12]. Although long noncoding RNAs do not play the role of coding proteins, they can regulate the expression and function of related genes at the RNA level through corresponding regulatory mechanisms [13]. Besides, in recent years, more and more studies focused on the prognostic value of long noncoding RNA, and many accurate lncRNA-based prediction models have been created and tested [14–16].

Uterine corpus endometrial carcinoma (UCEC) is a common gynaecological tumor, which occupies a major position in gynaecological tumor cases in developed countries [17], and it is still the second most common tumor in developing countries. It has been reported that there are an estimated 382000 new cases and 89900 deaths worldwide in 2018 [18]. Although surgical treatment provides a good prognosis for patients with early UCEC, the 5-year OS of patients with recurrent or metastatic UCEC is significantly lower [19]. Accurate prediction of individual prognosis is helpful to early identify patients with poor prognosis and individualized accurate treatment. Therefore, in this study, we devoted ourselves to identifying lncRNAs associated with the TP53 signaling pathway in UCEC and constructed prediction models based on these lncRNAs. At the same time, we further studied the potential relationship between this prediction model and immune microenvironment and drug sensitivity.

## 2. Materials and Methods

### 2.1. Patients and Row Data

528 UCEC patients with corresponding clinicopathological characteristics and sequencing data of 552 UCEC tumor samples and 35 normal samples were downloaded from the TCGA database (https://portal.gdc.cancer.gov/). Besides, as TP53 was one of the most mutated genes in UCEC, the mutation profiles of UCEC were also retrieved from the TCGA database. “KEGG TP53 signaling pathway” was searched and downloaded from MsigDb (https://www.gsea-msigdb.org/gsea/msigdb/).

### 2.2. TP53 Pathway in UCEC and Identification of TP53 Pathway-Related lncRNAs

First, we wondered whether the TP53 pathway is differentially activated between tumor samples and normal samples, and we performed gene set enrichment analysis (GSEA). Then we extracted the expression of genes in the TP53 signaling pathway, applied the Spearman correlation test between this expression atlas and lncRNA expression atlas. |Cor| > 0.5 and adjusted *p* value <0.05 were set as the threshold to define TP53 pathway-related lncRNAs [20].

### 2.3. Randomization and Signature Construction

We randomly divided all UCEC patients into training sets and test set at a ratio of 1 : 1, then performed univariate cox regression, LASSO regression, and multivariate cox regression in proper order for the final prognostic signature. Then, there established a risk formula according to the signature:

(1) $$\begin{array}{c} \text{Riskscore}=\overset{N}{\underset{i=1}{\sum }}\left(\text{Exp}\left(i\right)∙\text{coef}\left(i\right)\right), \end{array}$$

where *i* represents the *i*th TP53 pathway-related lncRNAs; *N* represents that there a total of *N* TP53 pathway-related lncRNAs in the prognostic signature; exp(*i*) represents the expression value of *i* (in FPKM format); coef(*i*) represents the coefficient of *i*. Then, all samples obtained a corresponding risk score, and we divided all samples into high-/low-risk groups according to the medium risk score in the training set.

### 2.4. Survival Analysis, ROC Curves, and Subgroup Analysis

We plot the survival curves by Kaplan-Meier methods in the training set, test set, and all samples. The log-rank test was used to investigate the survival differences between high-risk and low-risk groups. Notably, the ROC curves in the training set, test set, and all samples were assembled. Besides, the area under curves (AUC) at 1, 3, and 5 years was calculated to emphasize the prediction capability of the prognostic signature. Besides, we divided all patients into several subgroups according to their clinicopathological characteristics and performed survival analysis in each subgroup to explore whether this signature was accurate in all subgroups.

### 2.5. Interaction Network and Sankey Plot

We were interested in the interaction network between the TP53 pathway and these lncRNAs. Thus, we visualized the interaction network by Cytoscape (version 4.0.8) and then plot the Sankey plot to show the relationship and risk type of these lncRNAs.

### 2.6. Immune Infiltration, Drug Response, and Mutation Atlas

The CIBERSORT algorithm was carried out to emphasize the immune infiltration of each patient [21], and then we performed Wilcoxon tests to discover the differences in immune infiltration between high-risk and low-risk patients. Besides, R package “pRRophetic” was used to predict the drug response to cisplatin and paclitaxel [22]. Then, the drug response was also compared between high-risk and low-risk groups. Finally, as TP53 is one of the most mutated genes in UCEC, we sorted the mutation profiles according to the risk score and explored the differences in their mutation atlas.

## 3. Results

### 3.1. Characteristics of Patients Enrolled in This Study

A total of 528 patients with complete clinical information and transcriptional data were enrolled in this study and randomly split into a training set (*N* = 263) and test set (*N* = 265). Their clinicopathological characteristics were shown in Table 1, and it seems there were no baseline differences between the training set and test set. Notably, the races of patients with UCEC were consist of American Indian or Alaska Native, Asian, Black or African American, Native Hawaiian or other pacific islander, and White. Among of them, the White was the major race. The longest follow-up duration in this cohort were 18.79 years. And the pathological G-stage refers to the FIGO 1971 staging system. Besides, 16 of 528 UCEC patients received certain radiotherapy, and the radiotherapy history of the left 512 patients was unknown.

### 3.2. GSEA Analysis and Signature Construction

Firstly, we sorted the transcriptome matrix according to the tissue type that there was tumor tissue to normal tissue from left to the right. Then we input the “KEGG TP53 signaling pathway” as enriched pathway and carried out the GSEA analysis. Interestingly, we found TP53 signaling pathway was significantly enriched in the tumor samples (Figure 1(a), NES = 1.739, normalized *p* value =0.008), which indicated TP53 pathway was highly activated and played an essential role in UCEC. Following this, we performed Spearman correlation test between the expression value of genes in the TP53 signaling pathway and expression value of all the lncRNAs. Initially, we discovered 775 TP53 pathway-related lncRNAs with |Cor| > 0.5 and adjusted *p* value <0.05. Finally, we constructed a nine TP53 pathway-related lncRNA signature by univariate Cox regression, LASSO regression (Figures 1(b) and 1(c)), and multivariate Cox regression (Figure 1(d)) in order. The detailed coefficient of each lncRNA in this signature was showed in Table 2.

### 3.3. Survival Analysis and ROC Curves

This nine TP53-related lncRNAs signature showed great capability in the log-rank test in the training set (Figure 2(a), *p* < 0.001), test set (Figure 2(b), *p* < 0.001), and all samples (Figure 2(c), *p* < 0.001). Besides, this signature also showed stable AUC in predicting survival in training set (Figure 2(d), 1-year AUC = 0.777, 3-year AUC = 0.785, and 5-year AUC = 0.759), test set (Figure 2(e), 1-year AUC = 0.736, 3-year AUC = 0.618, and 5-year AUC = 0.657), and all samples (Figure 2(f), 1-year AUC = 0.760, 3-year AUC = 0.716, and 5-year AUC = 0.729). The distribution of risk score and survival status in each group was also shown in Figures 2(g)–2(i).

### 3.4. Interaction Network and Sankey Plot

We visualized the interaction network containing 10 mRNAs in the TP53 signaling pathway and these nine TP53-related lncRNAs as shown in Figure 3(a). Also, the Spearman correlation test was conducted between these 19 genes, and we found all the correlation was positively correlated (Figure 3(b)). The Sankey plot showed four protective lncRNAs and five risky lncRNAs in this signature (Figure 3(c)).

### 3.5. Immune Infiltration and Drug Response

The immune infiltration atlas of all patients between high-risk and low-risk groups was summarized in Figure 4(a). Here, we focused on the significant differential infiltrated immune cells containing M2 macrophages and activated dendritic cells (DC) that both activated DC and M2 macrophages were significantly higher infiltrated in high-risk patients than low-risk patients (Figures 4(b) and 4(c)). Besides, in the comparison of IC50 to the chemotherapy, the drug responses to both cisplatin and paclitaxel were significantly different between high-risk and low-risk patients that high-risk patients showed a more sensitive response to both cisplatin and paclitaxel (Figures 4(d) and 4(e)).

### 3.6. Mutation Atlas and Subgroup Analysis

Mutation atlas, including the 20 highest mutated genes in high-risk patients and low-risk patients, was shown in Figure 5(a) and Figure 5(b). The significant differential mutated genes were explored between high-risk and low-risk patients by *χ*^2^ test as shown in Table 3. Notably, TP53 mutation ranks the first in these differential mutation genes that showed a mutation proportion of 49% in high-risk patients and only 23% in low-risk patients (*p* < 0.001). Besides, this signature showed a great performance in all subgroups (Figures 5(c)–5(g)). In both patients with age > 65 (Figure 5(c), *n* = 228, p = 0.002) and patients with *age* ≤ 65 (Figure 5(d), *n* = 300, p =0.002) subgroups, this risk score is associated with the overall survival that patients with high-risk showed a poor OS. Besides, in all the subgroups of G-stage, including G1 subgroup (Figure 5(e), *n* = 98, *p* = 0.028), G2 subgroup (Figure 5(f), *n* = 120, *p* = 0.005), and G3 subgroup (Figure 5(g), *n* = 310, *p* = 0.027), this risk score is quite effective. All these results showed the universality and practicability of our prognostic signature.

## 4. Discussion

P53 is a tumor suppressor protein and transcription factor, which can regulate cell division, prevent DNA mutated or damaged cells from dividing and induce abnormal apoptosis of these DNA damaged cells by upregulating transcriptional apoptosis signals to prevent the formation of the tumor [23, 24]. It can respond to cell stress or DNA damage and activate different transcriptional targets. It is worth noting that p53 can coordinate various responses, including cell cycle arrest, DNA repair, metabolic changes, antioxidation, antiangiogenesis, autophagy, cellular senescence, and apoptosis [7]. Recent studies have also shown that TP53 is a significant iron death-inducing factor [25]. Therefore, the TP53 signaling pathway is crucial in the occurrence and development of tumors. It is necessary to study the new functions and new regulatory factors of TP53.

In this study, we first confirmed that the TP53 signaling pathway is highly activated in UCEC, then identified 775 TP53 signaling pathway-related lncRNAs, constructed a prognostic signature in the training set, and verified it in the test set. This prognostic signature shows high prediction accuracy in the training set, test set, all samples, and subgroups. More importantly, even though the prognosis of high-risk patients is worse, we found that they are more sensitive to cisplatin, which means that the patient differentiation of our prediction model can be used to assist clinical decision-making. Finally, we found significant differences in the infiltration of M2 macrophages between high-risk and low-risk patients, and the mutation rate of TP53 was higher in high-risk patients. In a word, we devote to identifying TP53 pathway-related lncRNAs in UCEC and established a nine TP53 pathway-related lncRNA signature. This signature has three main functions, and they are risk stratification, medication guidance, and mutation prediction. Higher risk score results in a poor prognosis but better response to the chemotherapy to cisplatin and paclitaxel, and a higher probability with mutant type of TP53.

The relationship between TP53 mutation and the tumor microenvironment has always been a controversial issue [26, 27]. Many studies have shown that TP53 mutation plays a negative role in antitumor immunity [26]. However, many studies have reported that TP53 mutation can promote antitumor immunity [28, 29]. In our study, high-risk patients were associated with significantly higher levels of M2 macrophage infiltration and activated DC cell infiltration. Although activated DC cells seem to present more tumor antigens or tumor neoantigens, M2 macrophages with a higher proportion of infiltration shape an anti-inflammatory and tumor-promoting immune microenvironment [30, 31], which also explains why patients with high-risk have a worse prognosis. Another interesting finding is the difference in sensitivity to cisplatin between patients with high- and low-risk. Traditional cytotoxic drugs usually play an antitumor role by blocking cell proliferation or inducing tumor cell apoptosis [32]. One of the most used chemotherapy regimen for endometrial cancer is the TC regimen: paclitaxel plus carboplatin [33]. Our study shows that high-risk patients are more sensitive to cisplatin and paclitaxel, which may be related to the difference in gene mutation spectrum in high-risk and low-risk patients.

Among these lncRNAs, *CFAP58-DT* has been reported associated with genome instability [34]. This is interesting and consistent with our study that TP53 is associated with genome instability, and we identified *CFAP58-DT* as a TP53 pathway-related lncRNA in UCEC. Also, Jin et al. identified *AC092794.1* as an immune-related lncRNA in lung adenocarcinoma [35]. Moreover, we found a significant difference in immune infiltration between high-risk and low-risk patients in the present study. All these verified the reliability of our results. However, there existed some limitations in this study. On the one hand, though we have examined this prognostic signature in the test set, it still needs a large sample, multicenter independent cohort for validation. On the other hand, we need to conduct more experiments in the laboratory to further verify the regulation or coexpression of these lncRNAs on the TP53 signaling pathway. Besides, there lacks detail pathological information of patients, which is critical for our comprehension of the association between TP53 related pathway, this signature, and the pathological stages and grades. And here, we predicted the individual response to the chemotherapy by the “Prophetic” algorithm, which can only predict the “IC50” of each patient to the chemotherapy, which might be more meaningful for clinicians if it can predict the response classifications such as complete response (CR), partial response (PR), and stable disease (SD).

In summary, we verified the significant role of TP53 signaling pathway in UCEC and constructed a critical TP53-related mRNA-lncRNA interaction network, which may provide potential therapeutic targets and biomarkers of companion diagnosis. More importantly, we identified a nine TP53 pathway-related lncRNA signature in UCEC and verified this prognostic signature in the test set. Besides, though high-risk patients showed a poor prognosis, they were more sensitive to the cisplatin and paclitaxel. The differential immune infiltration and mutation atlas associated with this signature need further investigation in the future.

## Figures and Tables

**Figure 1:** Signature construction. (a) Significantly enriched TP53 signaling pathway in tumor tissues. (b) Identification of TP53 pathway-related lncRNAs. (c) Variables going to zero as we increase the penalty (lambda) in the objective function of the LASSO. (d) 10-fold cross-validation for tuning parameter selection in the LASSO model, −5 < lambda. Min < −4.5. (e) A nine TP53 pathway-related lncRNA signature.

**Figure 2:** Validation of the signature. (a) Survival analysis in training set. (b) Survival analysis in test set. (c) Survival analysis in all patients. (d) ROC curves in training set. (e) ROC curves in test set. (f) ROC curves in all patients. (g) Risk plot in training set. (h) Risk plot in test set. (i) Risk plot in all patients.

**Figure 3:** Interaction network and Sankey plot. (a) TP53 pathway mRNA-TP53 pathway-related lncRNA interaction network. (b) Correlation circus plot. (c) Sankey plot.

**Figure 4:** Immune infiltration and drug response. (a) Summary of the immune infiltration in all patients with *p* < 0.05. (b) Differential infiltration of M2 macrophages between high-risk and low-risk patients. (c) Differential infiltration of active dendritic cells between high-risk and low-risk patients. (d) Drug response to cisplatin between high-risk and low-risk patients. (e) Drug response to paclitaxel between high-risk and low-risk patients.

**Figure 5:** Mutation atlas and subgroup analysis. (a) Mutation atlas of high-risk patients. (b) Mutation atlas of low-risk patients. (c) Survival analysis in patients with age > 65. (d) Survival analysis in patients with age ≤ 65. (e) Survival analysis in patients with G1. (f) Survival analysis in patients with G1. (g) Survival analysis in patients with G1.

**Table 1:** Characteristics of patients between train and test group.

Covariates	Type	Total (*n* = 528)	Test (*n* = 265)	Train (*n* = 263)	*P* value
Age	<=65	300 (56.82%)	149 (56.23%)	151 (57.41%)	0.8511
	>65	228 (43.18%)	116 (43.77%)	112 (42.59%)	

Grade	G1	98 (18.56%)	52 (19.62%)	46 (17.49%)	0.1579
	G2	120 (22.73%)	51 (19.25%)	69 (26.24%)	
	G3	310 (58.71%)	162 (61.13%)	148 (56.27%)	

**Table 2:** Coefficients of the risk model.

Id	Coef	HR	HR.95 L	HR.95H	*P* value
AC100830.1	1.913841073	6.779077787	2.273192433	20.21645637	0.000596999
AP000593.3	1.86348689	6.446174728	1.941979816	21.39732261	0.002332998
AC096586.2	-0.874282726	0.417161131	0.147995743	1.175867666	0.098217623
AL359220.1	-4.010417767	0.018125821	0.000115907	2.834565161	0.119760544
AC092953.2	1.020800007	2.775414226	1.080095651	7.13170553	0.034007797
CFAP58-DT	0.606034734	1.833148049	0.956095862	3.514743554	0.068034498
AC139887.1	-0.497802303	0.607865096	0.406569615	0.908823387	0.015272263
AC092794.1	-0.72260666	0.485485111	0.21107604	1.116639258	0.089062806
CDKN2A-DT	0.998649738	2.714613913	1.068732322	6.895205231	0.035752743

**Table 3:** Differential mutated genes between high-risk patients and low-risk patients.

Gene	H-wild	H-mutation	L-wild	L-mutation	*P* value
TP53	132 (50.97%)	127 (49.03%)	203 (76.89%)	61 (23.11%)	1.15E-09
PTEN	125 (48.26%)	134 (51.74%)	69 (26.14%)	195 (73.86%)	2.65E-07
ANKRD24	238 (91.89%)	21 (8.11%)	258 (97.73%)	6 (2.27%)	0.004835366
CTNNB1	210 (81.08%)	49 (18.92%)	186 (70.45%)	78 (29.55%)	0.006301608
ARID1A	160 (61.78%)	99 (38.22%)	132 (50%)	132 (50%)	0.008705329
CFAP221	238 (91.89%)	21 (8.11%)	257 (97.35%)	7 (2.65%)	0.009954249
DDX17	252 (97.3%)	7 (2.7%)	243 (92.05%)	21 (7.95%)	0.013382989
MAP3K1	237 (91.51%)	22 (8.49%)	222 (84.09%)	42 (15.91%)	0.014141527
NYNRIN	225 (86.87%)	34 (13.13%)	247 (93.56%)	17 (6.44%)	0.015083671
HK1	236 (91.12%)	23 (8.88%)	255 (96.59%)	9 (3.41%)	0.015193715
RACGAP1	239 (92.28%)	20 (7.72%)	257 (97.35%)	7 (2.65%)	0.015412168
POTEH	239 (92.28%)	20 (7.72%)	257 (97.35%)	7 (2.65%)	0.015412168
CTCF	207 (79.92%)	52 (20.08%)	186 (70.45%)	78 (29.55%)	0.016225864
GRIPAP1	251 (96.91%)	8 (3.09%)	242 (91.67%)	22 (8.33%)	0.016812212
HHIPL2	235 (90.73%)	24 (9.27%)	254 (96.21%)	10 (3.79%)	0.018105893
RERE	246 (94.98%)	13 (5.02%)	235 (89.02%)	29 (10.98%)	0.018824496
GJA8	252 (97.3%)	7 (2.7%)	244 (92.42%)	20 (7.58%)	0.020312746
MTIF2	250 (96.53%)	9 (3.47%)	241 (91.29%)	23 (8.71%)	0.020553208
SREBF2	250 (96.53%)	9 (3.47%)	241 (91.29%)	23 (8.71%)	0.020553208
SLC39A10	237 (91.51%)	22 (8.49%)	255 (96.59%)	9 (3.41%)	0.022779625
JPH3	236 (91.12%)	23 (8.88%)	254 (96.21%)	10 (3.79%)	0.026762318
ZNF786	250 (96.53%)	9 (3.47%)	242 (91.67%)	22 (8.33%)	0.030208582
ZNF644	230 (88.8%)	29 (11.2%)	249 (94.32%)	15 (5.68%)	0.034496492
INO80D	234 (90.35%)	25 (9.65%)	252 (95.45%)	12 (4.55%)	0.035123799
AGPAT9	251 (96.91%)	8 (3.09%)	244 (92.42%)	20 (7.58%)	0.037079599
KSR2	246 (94.98%)	13 (5.02%)	237 (89.77%)	27 (10.23%)	0.03788678
CLCA2	237 (91.51%)	22 (8.49%)	254 (96.21%)	10 (3.79%)	0.039129817
GANAB	248 (95.75%)	11 (4.25%)	240 (90.91%)	24 (9.09%)	0.041212025
ZNF610	240 (92.66%)	19 (7.34%)	256 (96.97%)	8 (3.03%)	0.042632701
SPZ1	240 (92.66%)	19 (7.34%)	256 (96.97%)	8 (3.03%)	0.042632701
PVRL3	240 (92.66%)	19 (7.34%)	256 (96.97%)	8 (3.03%)	0.042632701
C15orf39	250 (96.53%)	9 (3.47%)	243 (92.05%)	21 (7.95%)	0.04393845
EP300	234 (90.35%)	25 (9.65%)	222 (84.09%)	42 (15.91%)	0.04446505
DSG2	247 (95.37%)	12 (4.63%)	239 (90.53%)	25 (9.47%)	0.047003188
RHOBTB2	239 (92.28%)	20 (7.72%)	255 (96.59%)	9 (3.41%)	0.04955972
CHSY3	239 (92.28%)	20 (7.72%)	255 (96.59%)	9 (3.41%)	0.04955972
ITIH3	239 (92.28%)	20 (7.72%)	255 (96.59%)	9 (3.41%)	0.04955972

Note: H: High-risk patients, L: Low-risk patients.

## Data Availability

Source data of this study were available from corresponding author (email: hedeng2002@163.com).

## Abbreviations

UCEC: Uterine corpus endometrial carcinoma
lncRNA: Long noncoding RNA
Linc RNA: Long intergenic noncoding RNA
NAT: Natural antisense transcripts
LASSO: Least absolute shrinkage and selection operator.
